RETRACTED

# Successful management of massive intraoperative pulmonary fat embolism with percutaneous cardiopulmonary support

**DOI:** 10.4103/0972-5229.43684

**Published:** 2008

**Authors:** Suman Sarkar, Krutisundar Mandal, Prithwis Bhattacharya

**Affiliations:** **From:** Department of Anesthesiology, IMS Banaras Hindu University, Varanasi-221 105, Uttar Pradesh, India

**Keywords:** Fat embolism, orthopedic surgery, percutaneous cardiopulmonary support

## Abstract

We report a patient who sustained catastrophic pulmonary fat embolism, during open reduction, internal fixation (ORIF) of fracture femur' In our opinion, the use of percutaneous cardiopulmonary support with (PCPS), saved the patient from certain death.

## Introduction

Pulmonary fat embolism is a life-threatening complication for patients with long-bone fractures undergoing surgery.[1–4] The incidence of the fat embolism syndrome ranges between 0.9 and 2.2%, and the mortality rate has been reported to be 13-87%.[5–8] We report a patient with severe haemodynamic instability following fat embolism, who was successfully treated using percutaneous cardiopulmonary support (PCPS).

## Case Report

A 65 year old woman had a fall in her bathroom, and presented to the hospital with Fracture shaft of femur. She was admitted to hospital for repair of the left femur fracture. An ORIF with an intramedullary nail, was planned to repair the fracture. Intraoperatively basic monitoring with continuous ECG, non-invasive blood pressure, and pulse oximetry was carried out. The procedure was done with epidural anaesthesia, given in the lumbar region -L3-L4 space, using isobaric bupivacaine 0.5% (16ml). The patient was sedated using intermittent Midazolam 2 mg IV, and the patient received oxygen through a venti-mask. After epidural block her blood pressure was 110/64 mm Hg, heart rate was 83 / min, and the SpO_2_ was 99%. Approximately 15 min after the insertion of the intramedullary nail, the patient suddenly became restless and this excitement progressed to generalized seizures. The oxygen saturation decreased from 99 to 80%. The patient became tachypnoeic, and the ECG showed ventricular bigeminy. Within seconds, she developed profound hypotension and shock The oxygen saturation could not be recorded. The patient was immediately intubated with a 7.5 mm endotracheal tube and positive pressure ventilation commenced. The initial end tidal CO_2_ was noted to be between 0 and 2.02. An arterial line was inserted, and an arterial blood gas analysis obtained, which showed a pH 7.019 of pCO_2_ was 20.17 mmHg, and paO_2_ was 107.57 mm of Hg, with a base deficit of 3.6 meq litre while breathing 100% oxygen. We urged the surgeon to complete suturing the skin as soon as possible. While the surgeon was suturing the skin, we inserted a pulmonary artery (PA) catheter. The systolic pulmonary arterial pressure was 48 mm Hg and the diastolic pressure was 32 mm Hg. A Transthoracic echocardiogram revealed massive dilatation of the right ventricle, the diameter of the inferior vena cava was 26 mm, and diametric change accompanying respiration was not observed. The left ventricular function was normal. We diagnosed the cause for the circulatory collapse as due to acute right heart failure (acute cor pulmonale) The patient then developed atrial fibrillation and subsequently pulseless ventricular tachycardia and required defibrillation, and cardiopulmonary resuscitation. CPR was continued in the operating theatre. Blood gas analysis during CPR showed a pH 7.075 of pO_2 -_ 340.64 mm of Hg, and pCO_2 -_ 41.84 mm of Hg with a base deficit of 16.9 mEq litre while breathing 100% oxygen. The end-tidal carbon dioxide was between 0 and 12 mm of Hg, and oxygen saturation could not be monitored.

RETRACTED

After successful CPR using epinephrine, atropine, vasopressin, and debfibrillation, continuous infusion of Norepinephrine 2 µg / kg / min and Dobutamine 20 µg / kg / min were started and the rates of infusions were adjusted to maintain the arterial systolic blood pressure >80 mm Hg. Systolic PA pressure was 51 mm Hg and pulmonary capillary wedge pressure (PCWP) was 33 mm Hg. A repeat Transthoracic echocardiogram (TTE) showed that the right ventricle was severely dilated but left ventricular function was maintained. After about an hour of continuous resuscitation, despite optimal maximal doses of pharmacological support, we could not maintain the systolic blood pressure >80 mm Hg; at this stage, we decided to place a portable PCPS.

The PCPS is composed of heparin-coated circuits (Carmeda™ Closed Chest Support System), a biopump, a heat exchange unit, and a Maxima™ membrane oxygenator (Medtronic Cardiopulmonary CO, Anaheim, CA, USA). We inserted a 19 Fr drainage cannula into a femoral vein and 17 Fr re-infusion cannula into the femoral artery percutaneously. The initial blood flow was 2.5 litre min and the rotation rate of the biopump was 2500 rpm. The oxygen fraction was 1.0 at 4.0 litre min^-1^. About one hour after PCPS was started, the patient started showing signs of recovery, Her ECG returned to normal sinus rhythm and her circulatory failure began to improve, her systolic blood pressure was 92 mm Hg and her heart rate was between 90 - 100 beats / min. The PA pressure gradually decreased from 51 to 34 mm Hg, and her general condition became stable. The patient's blood gas analysis at this time showed a pH pH 7.34, pO2 of pO_2_ -477.34 mm of Hg, and pCO_2 -_ 27.74 mm of Hg with 100% oxygen. The mixed venous oxygen saturation increased from 48 to 75%. The blood flow was maintained at 2.5 litre min and her core temperature had been lowered to less than 34°C for the protection of cerebral function. After the initiation of PCPS and having stabilized her cardiovascular condition, we transferred the patient from the operating theatre to a radioscintigraphic examination room as by this time we had strong suspicion of fat embolism. The radioscintigram showed diffuse multiple defects of blood flow in both lungs. After scintigraphic examination, we brought the patient to the intensive care unit (ICU).

RETRACTED

We diagnosed the patient as having pulmonary fat embolism from the presence of lipid granules, sampled from the tip of the PA catheter and stained with oil red O.[9] On day one in ICU, the patient's condition was stable on PCPS. On day two, since the patient was cardiovascularly stable, we lowered the PCPS flow to 1.0 litre min and then to 0.5 litre min. Throughout this time, the systolic blood pressure was maintained above 120 mm Hg and her heart rate was between 80 - 90 beats/min. The cardiac output (CO) was more than 3.5 litre min. The PA pressure had been between 25 and 30 mm Hg. We therefore decided to stop and remove the PCPS from the patient. Immediately after disconnecting the drainage cannula from the femoral vein, the patient crashed and had a very low systolic blood pressure with the ECG showing wide QRS complexes. PCPS was resumed immediately. An echocardiogram showed dilatation of the right ventricle, septal akinesis, and hypo kinesis of the left ventricle and the LV ejection fraction was less than 10%. We therefore continued to support the patient on PCPS. We had to give more time for the recovery of her cardiac function. On day three in ICU, the patient;s CO was 4.0 litre min^-1^ and PCWP 20 mm Hg. On the fourth ICU day, the systolic blood pressure was 140 mm Hg, heart rate between 80 and 90 beats min, systolic PA pressure between 25 and 30 mm Hg, PCWP 20 mm Hg, and cardiac index 3.6 litre m^-2^ min using a PCPS flow of 1.0 litre min. IV digital subtraction angiography at this stage showed adequate blood supply to both the lungs, except for a small apical part of the left lung. Good wall motion of the heart was observed at the same time. PCPS was then stopped for 30 min and we confirmed that the patient's haemodynamic condition remained stable. We then proceeded to wean the patient off PCPS. When the PCPS drainage cannula was withdrawn from the femoral vein, the PA systolic pressure suddenly increased from 30 to 65 mm Hg. and the ECG showed paroxysmal supra-ventricular tachycardia with a heart rate between 180-190/ min. The arrhythmia was successfully treated with cardioversion. The systolic arterial blood pressure was between 100 and 120 mm Hg. However the PA pressure remained as high as 65 mm Hg and we administered Prostaglandin 0.5 µg / kg.

RETRACTED

After PGE_1_ infusion, the PA systolic pressure gradually decreased from 65 to 40 mm Hg. One hour after weaning from PCPS, the patient had a blood pressure of 120/90 mm Hg, 90-100 /min, cardiac index of 3.0 L/min, and mixed venous oxygen saturation of 73%. However, she continued to have high pulmonary pressures So we continued PGE_1_ at 0.2 µg / kg / min, which gradually relieved pulmonary hypertension and the PA pressure decreased to 25 mm Hg (mean).

On the tenth postoperative day, the patient's PA pressure was pressure was 33/15 mm Hg (mean 19 mm Hg) and PCWP was 10 mm Hg, so we discontinued the PGE_1_ infusion. Sedation was ceased and the patient gradually woke up and was obeying commands. She was extubated, and subsequently transferred to HDU and then shifted to the ward without neurological complications.

## Discussion

In this case report, soon after a clinical diagnosis of cardiovascular collapse due to acute right heart failure secondary to massive fat embolism was suspected, an urgent echocardiogram helped us support our diagnosis. We have then described the successful management of this patient with aggressive resuscitation along with the use of cardiopulmonary bypass.

It is known that increase in pulmonary arterial pressure and resistance induce right ventricular failure that may persist for several hours.[10,11] Subsequent right ventricular dilatation may result in septal shift resulting in a decrease in left ventricular filling volume, leading to low CO. High right ventricular end-diastolic pressure in addition to low systemic blood pressure results in ischaemia of the right ventricle, potentiating the vicious cycle of right ventricular depression, dysfunction, and death. In our patient we kept cardiac massage going for an hour. Conventional treatment for right ventricular dysfunction includes the use of pulmonary vasodilators, volume loading, use of inotropes / vasopressors, Mechanical circulatory support is indicated for patients with right heart failure who show no improvement in response to conventional therapy.[10–12]

PCPS is a powerful resuscitative tool that may be used to support patients with cardiac arrest and improve their survival.[12–14] PCPS is an extracorporeal life support that involves the continuous drainage of venous blood to a pump and membrane oxygenator and re-infusion to a major vein or artery. Venovenous support is the primary mode for respiratory failure, known as extracorporeal membrane oxygenation; this is primarily used in respiratory failure when improved oxygenation is the main goal Venoarterial bypass provides full support for both respiratory and cardiovascular failure and is called as PCPS in Japan. Venoarterial bypass involves accessing the right atrium or inferior vena cava for venous drainage and infusion into femoral artery; this type of support is used for patients who require cardiovascular support. PCPS can be used for patients with circulatory collapse and patients with damaged pulmonary circulation.

RETRACTED

PCPS drains blood from the right atrium, bypassing the right ventricle and pulmonary circulation, and oxygenated blood is returned to the systemic circulation. Therefore, we think the use of PCPS for patients with severe pulmonary embolism with catastrophic cardiopulmonary failure is worth considering in appropriate patients.,

The advantage of PCPS is that cannulation of the femoral vessels can be performed relatively quickly percutaneously. PCPS can be started within 15 min. The heparin-coated PCPS circuit can be used for the patients soon after surgery. The main complications of PCPS are hemorrhage, ischemia to lower legs, infection, and hemolysis. Arterial blood flow is mechanically returned into the femoral artery in the antegrade direction to spontaneous heart beat that increases the afterload of the left ventricle and might cause left ventricular dysfunction. Considering the limitation and complications during longer PCPS, we had tried rapid initial weaning from PCPS, but we should have continued the PCPS until we had confirmed the recovery of cardiac function as acknowledged on the fourth postoperative day. Administration of a large dose of PGE_1_ reduces the afterload of the right ventricle and improves refractory right heart failure. PGE_1_ is reported to be more pulmonary specific than Nitroglycerin, Sodium Nitroprusside, and Hydralazine, and resulted in the largest decrease in PA pressure.[15] PGE_1_ induced the largest decrease in PA pressure compared with the other pulmonary vasodilators Isoproterenol, Prostacyclin, and Nifedipine.[16] PCPS maintained our patient's condition well so that we did not use PGE_1_ while PCPS support was continued. However, retrospectively, we think we should have administered PGE_1_ from the start of the PCPS, then perhaps the cardiopulmonary status of the patient might have been stabilized better. If conventional pharmacological measures are not capable of stabilizing a patient with severe pulmonary fat embolism, PCPS is worth considering. This case shows that PCPS could provide effective support for the patients with fatal pulmonary fat embolism syndrome. Administration of PGE_1_ seemed effective for PH after weaning from the PCPS support.
